# The interplay of phenotype and genotype in *Cryptococcus neoformans* disease

**DOI:** 10.1042/BSR20190337

**Published:** 2020-10-16

**Authors:** Sophie Altamirano, Katrina M. Jackson, Kirsten Nielsen

**Affiliations:** Department of Microbiology and Immunology, University of Minnesota, Minneapolis, MN, U.S.A.

**Keywords:** Cryptococcus neoformans, genotype, microevolution, phenotype

## Abstract

*Cryptococcus neoformans* is an opportunistic fungal pathogen that causes life-threatening meningitis primarily in immunocompromised individuals. In order to survive and proliferate during infection, *C. neoformans* must adapt to a variety of stresses it encounters within the host. Patient outcome depends on the interaction between the pathogen and the host. Understanding the mechanisms that *C. neoformans* uses to facilitate adaptation to the host and promote pathogenesis is necessary to better predict disease severity and establish proper treatment. Several virulence phenotypes have been characterized in *C. neoformans*, but the field still lacks a complete understanding of how genotype and phenotype contribute to clinical outcome. Furthermore, while it is known that *C. neoformans* genotype impacts patient outcome, the mechanisms remain unknown. This lack of understanding may be due to the genetic heterogeneity of *C. neoformans* and the extensive phenotypic variation observed between and within isolates during infection. In this review, we summarize the current understanding of how the various genotypes and phenotypes observed in *C. neoformans* correlate with human disease progression in the context of patient outcome and recurrence. We also postulate the mechanisms underlying the genetic and phenotypic changes that occur *in vivo* to promote rapid adaptation in the host.

## Introduction

When it was first described in 1894, *Cryptococcus neoformans* was assumed to be a single species. More than a century of work, however, has revealed that what is now referred to as the *Cryptococcus* sp. complex has notable heterogeneity in pathogenesis, genetics, epidemiology, ecology, and biochemistry. Instead of the single species described in 1894, we now know that the *Cryptococcus* sp. complex contains at least seven distinct species or two major species complexes [1,2]. The *Cryptococcus* sp. are able to cause disease in both immunocompromised and immunocompetent individuals, although disease is much more commonly observed in the immunocompromised. Individuals at greatest risk of developing disease are those living with HIV/AIDS, patients taking corticosteroids, patients undergoing cancer chemotherapy, solid-organ transplant recipients, or individuals with other causes of immune deficiency [3]. Infection occurs when a person inhales a *Cryptococcus* spore into the lungs. If this initial infection is not eradicated by the immune response, or controlled in the lungs via granuloma formation, the infection can progress to result in fungal pneumonia. Systemic dissemination can result in skin lesions, but the most common disease presentation is dissemination to the brain and subsequent cryptococcal meningitis [4]. If left untreated, cryptococcal meningitis is fatal. Recent research has indicated the important role *Cryptococcus* sp. genetics and cell phenotype play during interactions with the host to promote disease. This review highlights the need to define the interplay between genetics and phenotype to understand and prevent *C. neoformans* disease.

## Genetic variation affects patient disease outcomes

### How has our understanding of *Cryptococcus* genetics evolved?

The first indication that *Cryptococcus* was not a single species was the discovery that there were strain-specific differences to reactive antibodies. Yeast cells were found to consistently fit within one of four distinct serotypes: A, B, C, or D, based on antigenic differences in capsular polysaccharides [5,6]. Later work revealed that A and D serotypes had the ability to mate as did B and C, suggesting that *Cryptococcus* contained two species [7–9]. This theory was supported by additional work that showed the A, D and B, C serotypes had distinct ecology, epidemiology, biochemistry, and genomic structure [10–17]. Serotypes A, D were renamed *C. neoformans* var. *neoformans* and serotypes B, C named *C. neoformans* var. *gattii*. The next shift in nomenclature came as a result of the molecular age. Due to variations in the *URA5* gene that further differentiated serotypes A and D, serotype A was renamed *C. neoformans* var. *grubii* [18].

*C. neoformans* var. *gattii* was raised to the species level and eventually renamed *C. gattii* [10,19]. Additional molecular characterization of *C. gattii* populations revealed a substructure within the population and led to further subdivision into five species: *C. tetragatii, C deuterogattii, C. decagattii, C. bacillisporus*, and *C. gattii* [1]. This further subdivision of *C. gattii* has not been universally accepted by the research community with some researchers opting to use ‘*C. gattii* species complex’ to describe the complex population structure within *C. gattii* [2,20]. Concomitant with the renaming of the *C. gattii* species complex in 2015, *C. neoformans* var. *grubii* was renamed *C. neoformans* to reflect the fact that 95% of cryptococcal infections are caused by these strains, and *C. neoformans* var. *neoformans* was renamed *C. deneoformans* because these are the historical serotype D strains [1]. This name change was more universally accepted by the research community, and is used in this review, although ‘*C. neoformans* species complex’ is also commonly used (Figure 1A) [2].

**Figure 1:** Pathogenic *Cryptococcus* species Relatedness of the (**A**) *Cryptococcus* species complex and (**B**) subpopulations within *C. neoformans.* (A) There are five proposed species in the *C. gattii* species complex (yellow), and two species in the *C. neoformans* species complex (blue) [1,2,20]. (B) There are three evolutionarily distinct subpopulations within *C. neoformans*, as defined by molecular type: VNI, VNII, and VNB. VNII is very rarely found in clinical isolates. VNB is more diverse, was initially discovered in Botswana, and patients infected with these strains tend to have poor clinical outcomes. VNI causes the most cases of cryptococcosis and has three evolutionarily distinct subpopulations; ST93 and ST5 are in separate subpopulations [21,54,55].

Interestingly, the dominant clades VNI, VNII, and VNB observed in *C. neoformans* have not changed significantly as the field transitioned from the early microsatellite genotyping technologies to modern sequence-based technologies such as multilocus sequence typing (MLST) and whole-genome sequencing (WGS). The vast majority of clinical isolates are in the VNI clade (Figure 1B). The VNI and VNII clades are both globally distributed and tend to have predominantly clonal population structures [21–23]. In contrast, the VNB clade is primarily found in sub-Saharan Africa and South America and is highly diverse, suggesting ongoing or recent recombination [21,24]. To further classify major sequence types (STs) within the *C. neoformans* clades, a standardized, globally accepted MLST scheme for *C. neoformans* that uses seven unlinked genetic loci (*CAP59, GPD1, LAC1, PLB1, SOD1, URA5, IGS1*) sequenced individually or derived from WGS was developed [25]. Four of these genes are believed to be under neutral selective pressure, while three (*CAP59, LAC1*, and *PLB1*) code for *Cryptococcus* virulence factors. This globally accepted method to identify the ST cluster of strains has begun to reveal the vast genetic diversity within *C. neoformans* and has also led to fine-scale studies associating *C. neoformans* genetics with geographic location and human disease.

### Are there differences in *Cryptococcus* sp. disease presentation?

The *Cryptococcus* sp. have dramatic differences in their ecology and disease epidemiology. *C. neoformans* and *C. deneoformans* predominantly cause disease in immunocompromised individuals across the globe, and thus are thought to be ubiquitous in the environment. *C. neoformans* causes 95% of all cryptococcal meningitis globally, and 99% of cryptococcosis cases in HIV/AIDS patients (Figure 2A) [4]. *C. neoformans* is known to be a disease of immunocompromised patients, but approximately 25% of patients with *C. neoformans* have no immunocompromising conditions (Figure 2B) [26–32]. In contrast, infections caused by strains in the *C. gattii* species complex are more commonly seen in immunocompetent individuals (∼64%) (Figure 2B) [30,31,33–36]. *C. gattii* infections had previously only been observed in tropical and subtropical regions of the world, leading to the assumption that *C. gattii* was ecologically restricted to these regions. However, an outbreak on Vancouver Island in Canada in 1999, that spread across North America, showed this assumption was incorrect [37]. Genetic analysis of the *C. gattii* outbreak strains revealed introgression of a ‘virulent’ South American genotype into previously uncharacterized ‘native’ North American genotypes, suggesting *C. gattii* was present previously in North America but was not associated with disease [38].

**Figure 2:** Epidemiology and pathobiology of the *Cryptococcus* species complex (**A**) *C. neoformans* is the most common species of *Cryptococcus* to cause infections globally, accounting for 95% of infections, compared with *C. deneoformans* (4%) and the *C. gattii* species complex (<1%) (left). In HIV+ patients, *C. neoformans* causes more than 99% of cases globally (right) [4]. (**B**) Infections by the *C. gattii* species complex most commonly occur in immunocompetent patients (64.3%), while infections by *C. neoformans* species complex primarily occur in patients with an immunocompromising condition (75%) [26–36]. (**C**) The most common clinical manifestations of cryptococcosis are skin lesions, pneumonia, and meningitis. Skin lesions, while rare, occur most often in patients infected with *C. deneoformans*, in approximately 14% of infections [41]. Patients with *C. neoformans* infections have skin lesions in 5% of cryptococcal meningitis cases [44]. Only 3% of *C. gattii* species complex cases have cutaneous cryptococcosis as a symptom [3]. The second most common manifestation of cryptococcosis is pneumonia. Pneumonia occurs most frequently in infections caused by *C. gattii* species complex infections, with 54% of *C. gattii* patients in the United States displaying lung involvement [36,45]. Species in the *C. neoformans* species complex manifest pulmonary cryptococcosis in 35% of clinical infections [41]. Cryptococcal meningitis occurs most frequently in the *C. neoformans* species complex, with over 80% of patients displaying meningitis symptoms [42]. Cryptococcal meningitis is less common in the *C. gattii* species complex with only 49% of patients in the United States developing meningitis [36].

Differences in disease progression between the *Cryptococcus* sp. are also observed in both patient populations and animal models. As mentioned, *C. neoformans* is known to be associated with cryptococcal meningitis in patients and readily disseminates to the brain after inhalation in mouse models of disease [39]. While not universal, *C. deneoformans* is often less virulent in animal models and less commonly observed as meningitis in clinical isolates worldwide (Figure 2C) [40–42]. *C. deneoformans* is more frequently found to cause disease in Europe, although many of these isolates have been shown to be hybrids with *C. neoformans* [43]. *C. deneoformans* also causes skin lesions more frequently; 14% of *C. deneoformans* patients manifest lesions, while skin lesions appear in 5% of *C. neoformans* patients and 3% of *C. gattii* patients (Figure 2C) [3,41,44]. The *C. gattii* species complex tends to cause a much more pronounced pneumonia in humans, and some studies have recapitulated this phenomenon in the animal model [45]. *C. gattii* manifests as pneumonia in 54% of patients in the United States (a percentage lower than patients in British Columbia), while the *C. neoformans* sp. complex causes pneumonia in 35% of cases (Figure 2C) [36,41,45]. Due to the known differences in *Cryptococcus* sp. disease potential and presentation and the fact that *C. neoformans* causes 95% of all cryptococcal meningitis worldwide, the following sections of this review will focus on *C. neoformans*.

### How does *C. neoformans* genotype impact patient outcome?

Cryptococcal meningitis mortality rates differ across the globe [46]. Historically, these differences have been attributed to treatment regimens, type of care, level of patient immune function, and patient genetics [47]. It was not until 2012, when Wiesner et al. published the first study linking the genetics of *C. neoformans* with virulence in humans, that the importance of *C. neoformans* genetics in virulence began to surface [48]. Wiesner et al. performed MLST sequencing on clinical isolates of *C. neoformans* from Ugandan HIV/AIDS patients and showed the isolates grouped into three distinct, phylogenetically linked clonal clusters within the VNI clade. In one cluster centered on ST5 and ST63 only 38% of the patients died, compared with a 79% mortality rate in the other two clusters, centered on ST93 and ST77, respectively (Figure 1B) [48]. Surprisingly, the differences in patient mortality were not due to numbers of yeast cells cultured from patient samples but rather alterations in the host immune response to the different genotypes that were associated with capsule and melanin production [48]. These data indicated for the first time that the pathophysiology of cryptococcal meningitis was associated with pathogen genotype within *C. neoformans*.

There have been several additional studies linking human disease with sequencing type. Beale et al. genotyped clinical isolates from South African HIV/AIDS patients using MLST [49]. This population exhibited much higher diversity than the Ugandan population, yet the authors still found that VNB and ST32 isolates both had worse patient outcome that could not be explained by *in vitro* phenotypic differences [49]. A study in Brazil that combined analysis of environmental and clinical isolates, and HIV/AIDS and transplant patients, showed that STs other than ST93 had lower patient survival rates, but ST93 was also over-represented in the environmental isolates (Figure 1B) [23,24]. In a study of renal transplant recipients in Brazil, patients infected with VNII were more likely to survive (Figure 1B) [50]. A particularly interesting link between patient disease and genotype was found in Asia, where *C. neoformans* infections are observed in immunocompetent individuals [51]. In Vietnam, analysis of isolates from immunocompetent patients showed that almost all are in a closely related VNI cluster centered on ST5 (Figure 1B) [52–54]. ST5 caused 82% of infections in HIV uninfected patients, compared with only 35% in HIV infected patients [26]. Combined, these studies analyzing clinical isolates from across the globe indicate that *C. neoformans* genotype is responsible for variations in patient clinical outcome but also highlight the global genetic diversity present in *C. neoformans*. In addition, the genetic changes in *C. neoformans* are occurring on too fine a level for the underlying mechanism to be defined by MLST or current *in vitro* assays. This showcases the need for WGS studies and better understanding of the host–pathogen interaction to truly link *C. neoformans* genetics with patient clinical outcome.

The first WGS studies in *C. neoformans* linked to clinical outcomes have provided unexpected results. Day et al. performed WGS on eight of the ST5 isolates mentioned previously [26]. The isolates were compared with the *C. neoformans* H99 reference genome and SNPs and INDELs either specific to the Vietnamese ST5 or non-ST5 isolates that caused translation truncation (and therefore, likely impacted protein production) were identified. The variants specific to ST5 were associated with 19 genes. Only three coded for previously identified virulence proteins. The non-ST5 variants truncated the translation of 25 genes, of which only 4 were previously known virulence determinants [26]. The next WGS study that investigated the link between *C. neoformans* genotype and patient phenotype was published in 2019 and specifically explored differences between ST93 isolates causing changes to patient outcome. Gerstein et al. performed WGS on clinical isolates from patients in Uganda, where ST93 is the most frequently identified sequence type [55]. They identified non-synonymous INDELs and SNPs that were specific to ST93 and not located in the extreme telomeric or centromeric regions. They then performed a genome-wide association study (GWAS) to explore association of the variants with patient clinical data that included parameters such as clinical outcome, patient immune response, and isolate *in vitro* phenotype. The GWAS identified 145 variants associated with 40 genes, with only two previously known to be virulence determinants. Gerstein et al. identified that four of these genes were novel virulence factors by testing deletion strains in a mouse inhalation model [55]. Perhaps most intriguing, considering the evolutionary distance between ST5 and ST93 (Figure 1B), is that four genes (*CNAG_ 05185, CNAG_05987, CNAG_02475*, and *CNAG_05185*) were identical between the two studies and an additional three were only a single gene off (*CNAG_07704, CNAG_04921, CNAG_01240* versus *CNAG_07703, CNAG_04922, CNAG_01241* for Day et al. and Gerstein et al., respectively). While genomic studies looking at the specific genetic polymorphisms that underlie the clinical difference between *C. neoformans* STs are still in their infancy, a number of striking observations can be made. First, while the exact polymorphisms within distinct ST lineages may differ, the observation that the same genes or regions of the genome are under selective pressure suggests these genes are universally important for *C. neoformans* virulence in humans. Second, only a small proportion of the virulence determinants identified in the GWASs had been previously identified as *C. neoformans* virulence factors. These data suggest that previous *in vitro* and *in vivo* studies aimed at defining the minimum requirements for *C. neoformans* to be a pathogen, which are shared by all the *Cryptococcus* sp*.*, may have missed the nuances of the host–pathogen interaction that impact clinical outcome in patients with cryptococcal meningitis. Thus, renewed effort needs to be placed on understanding the complexities of the *C. neoformans*–host interaction and how genetic polymorphisms impact these interactions.

## *C. neoformans* phenotypic variation affects patient disease outcomes

### What phenotypes occur *in vivo*?

In response to the host environment, pathogens often alter their morphology through changes in gene expression. These changes are associated with adaptation and survival in the host and are classified as ‘virulence’ phenotypes or factors. The transition to the host environment elicits two types of virulence associated phenotypic changes in *C. neoformans*: cell surface changes and cell size changes (Figure 3). Alterations to the cell surface include production of a polysaccharide capsule, modifications to the composition of the cell wall, and melanin synthesis. More recently, cell size changes have been recognized as important virulence phenotypes in *C. neoformans*. Distinct cell size phenotypes include the typical yeast cells, the large titan cells, and the small micro and titanide cells. Both cell surface and size modifications impact the host–pathogen interaction, but how these traits are impacted by genetic polymorphisms has yet to be explored.

**Figure 3:** Cell surface alterations and cell size changes in *C. neoformans* Model illustrating the cell surface alterations and cell size phenotypes in *C. neoformans*. The outside of the *C. neoformans* cell consists of a cell wall (highlighted in pink) and polysaccharide capsule. Typical cells (5–7 μm in diameter) have a capsule predominantly composed of GXM and GalXM (orange box). The cell wall of typical cells contains chitin, chitosan, α-glucan, melanin, and β-glucan (left pink box). Titan cells (>10 μm in diameter) exhibit a thickened cell wall with an increase in chitin, decreased glucan, and a layer of mannan (right pink box) [59]. Micro cells (<1 μm in diameter) also display thickened cell walls [66]. Titanides are 2–4 μm in diameter and are oval in shape. The cell wall of titanides are thinner than typical cells [71]. Abbreviations: GXM, glucuronoxylomannan; GXMGal, glucuronoxylomannogalactin.

Cell surface changes have long been known to be major virulence determinants in *C. neoformans*. Because mammalian cells do not have cell walls, the immune system uses sensing of many of the components of the fungal cell wall, such as β-glucan and chitin, to trigger the immune response to fungal pathogens. In response to the host environment, *C. neoformans* produces a polysaccharide capsule that is anchored to the exterior surface of the cell wall and is primarily made up of glucuronoxylomannan (GXM) and glucuronoxylomannogalactin (GXMGal) (Figure 3). The capsule is thought to help prevent recognition of the cell wall by the immune system. It undergoes size and structural alterations *in vivo* that result in antigenic variability [56]. Capsule is also shed from the surface of the cell, and this shed capsule has independent immune modulatory functions [57,58]. Recent studies show the *C. neoformans* cell wall also undergoes dramatic remodeling in response to the host environment [59]. The cell wall consists primarily of α-glucan, β-glucan, chitin, and chitosan (Figure 3). In the host the amount of β-glucan in the cell wall is reduced, while chitin increases, possibly utilizing chitosan to facilitate this process [59,60]. Melanin is also deposited into the cell wall and plays a protective role during infection, likely through detoxification of free radicals generated by the immune response [61]. Cell wall integrity appears to be important throughout this process, likely for cell survival and proper capsule formation [62,63].

In addition to cell surface alterations, *C. neoformans* also undergoes cell size variation *in vivo*. When grown *in vitro, C. neoformans* is typically 5–7 µm in diameter. During a murine pulmonary infection, cells with diameters ranging from smaller than 1 µm to as large as 100 µm have been observed [64–66]. Cells that exhibit an enlarged phenotype, defined as a cell diameter greater than 10 µm, are referred to as titan cells [64,65]. The characterization of titan cells has largely been confined to mouse models, but titan cells have also been observed in human infections [67–69]. Cells that exhibit a decreased size were first described in a murine pulmonary infection and are known as micro cells. Micro cells are <1 µm in diameter and little is known about this population of cells [66,70]. Interestingly, Dambuza et al. recently described a second population of small cells, known as titanides [71]. Titanides are 2–4 µm in diameter and oval in morphology. Titanides are associated with *in vitro* titan inducing conditions and are yet to be observed *in vivo* [71]. In addition to their distinct cell sizes, all these cell populations also display cell surface alterations (Figure 3). Titan cells have a thickened cell wall with a mannan layer and a highly cross-linked capsule [64,65]. Micro cells also display a thickened cell wall, while titanides have a thinner cell wall [66,71]. Cell size appears to vary by site of infection. Cells collected from the lungs of mice exhibit larger capsules and larger cell body diameters, while cells isolated from the brain exhibit smaller capsules and cell body diameters [58,72,73]. This organ-dependent size variation has also been described in human infections. Histology sections of postmortem brain contained significantly smaller cryptococcal cells and capsules than histology sections of postmortem lung [74]. Cell size variation may be important during infection as different cell sizes may be beneficial at different stages of infection. For instance, smaller cells may promote dissemination and survival within macrophages, while larger cells may aid in pathogen survival during pulmonary infection. Consistent with this idea, titan cells are primarily found in the lungs and have been shown to promote pathogenesis through decreased rates of phagocytosis and increased stress tolerance [64,75,76].

In addition to factors associated with cell surface and size, additional virulence factors including growth at 37°C, urease and phospholipase production, sphingolipid utilization, among others have been identified as major virulence factors. Extensive efforts to identify *in vitro* phenotypes, genes important to their formation, and subsequent mutant analysis—primarily using murine models—has been undertaken. For more information on these studies of virulence factor phenotypes in *C. neoformans*, and how they promote pathogenesis, please refer to the following reviews [77–80]. The analysis of virulence phenotypes has largely been confined to *in vitro* studies and animal models, but changes in virulence phenotypes may be responsible for differences observed in patient outcomes between clinical isolates.

### How does *C. neoformans* phenotype impact patient outcome?

Although there has been evidence of capsule enlargement, melanin synthesis, and titan cell formation during human infections, the extent of the phenotypic changes that occur in *C. neoformans* during human infection is largely unknown [61,67–69,81]. It is also unknown how these phenotypic changes may ultimately affect patient outcome and if they could be used as reliable indicators for patient outcome. However, within the last decade, progress has been made to better understand how *C. neoformans* phenotype relates to patient outcome in the context of human disease. Phenotypic analysis of clinical isolates isolated from the cerebrospinal fluid (CSF) of patients with significant disease paired with known clinical parameters has allowed for better understanding of the association of *C. neoformans* phenotype to patient outcome.

Recent studies have begun to investigate the correlation between human disease progression and *C. neoformans* cell surface changes using clinical data and virulence factor analysis of clinical isolates [81–88]. Several studies observed a significant correlation between capsule size and strain virulence [81–83]. Clancy et al. observed strains that produced smaller *in vivo* capsule size in mice were also more likely to have a higher lethal dose for 50% of mice (LD_50_) [82]. Interestingly, the correlation between LD_50_ and capsule size was not observed with *in vitro* induced capsule size [82]. Robertson et al. similarly showed that *ex vivo* capsule from human CSF samples correlated with several clinical parameters, including increased intracranial pressure and slower rate of fungal clearance [81]. This study also noted lack of correlation with *ex vivo* capsule and *in vitro* induced capsule formation [81]. Additionally, in the previously mentioned Wiesner et al. MLST study, strains associated with higher patient mortality displayed increased capsule shedding or melanin production [48]. Interestingly, the association with capsule shedding and patient mortality in the present study was not detected *in vivo* at time of patient diagnosis but rather associated with *in vitro* capsule shedding [48]. In contrast with these studies, Mukaremera et al. found no association between *in vivo* or *in vitro* capsule size and virulence in the mouse model [84]. The lack of agreement on the importance of the capsule to virulence throughout studies may be due to the different methodologies used to assess capsule size between studies. Typical *in vitro* capsule induction assays may not be sufficient to accurately evaluate the capsule formation of an isolate during human infection [81,82].

The phenotypic analysis of clinical isolates has largely focused on easy to measure virulence phenotypes such as *in vitro* capsule enlargement and/or shedding, melanin synthesis, growth at 37°C, urease activity, and phospholipase activity [77,85]. Several studies did not find a direct link between patient outcome and the virulence factors tested, especially with the use of *in vitro* assays [81–84,86–88]. Overall, these studies did highlight the high level of virulence factor heterogeneity between clinical isolates and the lack of association between a single virulence phenotype in determining disease outcome. Instead, a combination of multiple virulence phenotypes is likely to contribute to patient outcome.

Interestingly, two studies that incorporated analysis beyond the major cell surface virulence phenotypes showed the rate of *in vitro* phagocytosis was associated with patient mortality [86,88]. Alanio et al. showed isolates with high rates of *in vitro* phagocytosis and high intracellular proliferation displayed a higher risk of patient mortality [88]. A subsequent study by Sabiiti et al. similarly showed that increased rates of *in vitro* phagocytosis correlated with increased risk of mortality at 10 weeks post-diagnosis [86]. This study went on to show that isolates with increased rates of *in vitro* phagocytosis also displayed an increase in initial baseline fungal burden and increased laccase activity, indirectly suggesting a role for melanin in phagocytosis [86]. These studies show it may be necessary to go beyond the previously described virulence factors to better understand how the relationship between *C. neoformans* cell surface changes and host cell interactions impacts patient outcome.

In addition to phenotypic changes between isolates, it is important to note that *C. neoformans* also displays a wide range of phenotypes within a single population throughout the course of infection [66,70,89–92]. Phenotypic variation within an isolate may allow for rapid adaptation to the various host niches encountered during infection, suggesting the degree of phenotypic plasticity displayed by an isolate may also contribute to its virulence and the differences seen in disease outcome between isolates. A recent study investigating the size variability across clinical isolates from Botswana showed a correlation between size phenotype and clinical markers [70]. ‘Small’ phenotypes, which included micro cells and shed capsule, were found to be associated with clinical parameters important during later stages of infection, while ‘large’ phenotypes, which included increase in cell diameter and capsule size, were found to be associated with clinical parameters important during earlier stages of infection. Isolates typically exhibited either ‘large’ or ‘small’ phenotypes but rarely exhibited both. Interestingly, the four isolates that exhibited both ‘small’ and ‘large’ phenotypes all resulted in patient death [70]. Additionally, Thanh et al. showed clinical isolates able to infect immunocompetent patients displayed a significant increase in within-strain variation with regard to capsule and cell size [83]. These studies provide support to the idea that phenotypic heterogeneity within a population may contribute to host adaptation, which may subsequently impact patient survival. Similarly, Mukaremera et al. suggested that a single virulence factor would not dominate in *C. neoformans*, but rather the ability of an isolate to overcome a wider variety of stresses may result in increased virulence [84]. Thus, a strain’s ability to adapt to the host may be critical to disease outcome.

## Microevolution

### Does microevolution of *C. neoformans* occur during human infections?

Microevolution refers to rapid changes over a short period of time. During microevolution, selection of genetic and phenotypic alterations that allow for increased fitness occurs. There is evidence of microevolution in *C. neoformans* during passage in the lab, murine infection, and human infection [91,93–103]. The study of *C. neoformans* microevolution has primarily focused on recurrent infections in humans. Changes in karyotypes between recurrent isolates from humans result in altered virulence in a murine model [102–104]. The use of WGS coupled with phenotypic analyses has allowed for the identification of more specific genetic differences to be observed between initial and recurrent isolates and the phenotypic changes underlying these genetic changes to be assessed [99,101]. The genetic changes in recurrent isolates correlated with increased fluconazole resistance, and a smaller fraction correlated with other virulence phenotypes [101]. Exploring the genetic and phenotypic changes in recurrent human isolates collected from the CSF allows for better insight into the adaptations specific to the central nervous system. The changes in *C. neoformans* important for adaptation earlier in infection, such as establishment and progression of pulmonary infection, are yet to be explored in human samples. In a murine model, microevolution is thought to be organ dependent, and distinct subpopulations arise during a pulmonary infection, highlighting the heterogeneous initial response to the host environment [97,105]. The role each of these subpopulations plays during infection is unknown. Of particular interest is the population thought to be dormant cells [105]. Dormant cells may be important in host adaptation and reactivation of latent infections. There is epidemiological evidence of reactivation of dormant cells in human infections, but the characterization of dormant cells and their role in microevolution are yet to be assessed in clinical isolates [106].

### What are the possible mechanisms underlying microevolution in *C. neoformans*?

Genetic and phenotypic analyses of serial isolates from recurrent infections has provided insight into the genetic changes and subsequent phenotypic changes that occur during human infections that may promote host adaptation [99,101]. Although we now have a better understanding of the genetic and phenotypic changes *C. neoformans* undergoes during human infections, the mechanisms underlying these changes are still largely unexplored. In this section, we discuss the possible mechanisms that may promote microevolution in the human host, focusing on those that produce genetic alterations. The possible mechanisms discussed in this section include transposable elements (TEs), mutators, and titan cells (Figure 4).

**Figure 4:** Mechanisms of *in vivo* microevolution Model displaying possible mechanisms underlying the genetic and subsequent phenotypic changes seen during infection. Individual chromosomes are shown in black, and phenotype changes are represented by change in cell color. (**A**) During infection, TEs move throughout the genome. Transposon insertion into genes that may result in a range of phenotypes [111]. (**B**) Mutations in the MMR pathway result in cells with a higher rate of mutations (yellow stars) that may display various phenotypes [114,116]. (**C**) Polyploid titan cells undergo a reductive division to produce progeny with reduced genome sizes and genomic alterations, including cells with various whole chromosome aneuploidies (purple and green cells). Phenotype changes have also been observed in titan progeny that have no identified genomic alterations (tan cell) [76]. Abbreviation: MMR, mismatch repair.

TEs, or transposons, are segments of DNA that can move throughout the genome of an organism. TEs can independently proliferate, either by encoding their own enzymes for transposition or though reverse transcription (retrotransposons). TEs are common in eukaryotes and make up 5% of the *C. neoformans* genome, where they preferentially cluster on each chromosome into 40–100 kb regions near the centromere [95]. TEs can create or reverse mutations and cause changes in gene expression or regulation. As TEs can negatively disrupt the genome, most eukaryotes have evolved methods to defend against TE-induced mutagenesis. *C. neoformans* uses endogenously produced small RNAs (endo-siRNA) to silence TEs [107–110]. While limiting transposon mobilization to prevent detrimental mutagenesis is important under normal conditions, when adapting to a new, high-stress environment, transposons may prove beneficial. Since TEs are found in the *C. neoformans* genome and do contribute to mutagenesis, it is a logical hypothesis that TEs are involved in *C. neoformans* adaptation to the host through genetic and subsequent phenotypic alterations (Figure 4A). A recent paper analyzing transposons in *C. deneoformans* found an increase in TE activation when cells were grown at 37°C [111]. This same study hinted that a similar phenomenon exists in *C. neoformans*, where transposon activation during infection may act as a mechanism for microevolution (Figure 4A).

Mutators, or isolates that mutate rapidly under stress, have been identified in many species of fungi. Mutation phenotypes in *Saccharomyces cerevisiae, C. gattii*, and *C. neoformans* have been found to occur due to mutations in the mismatch repair (MMR) pathway, particularly in the MMR gene *MSH2* [112–114]. Mutations in genes involved in the MMR pathway of *C. neoformans—MSH2, MLH1*, and *PMS1*—result in isolates that showed a change in lung proliferation, suggesting a role in virulence [115]. Naturally arising mutations in these same three genes cause a mutator phenotype [114,116]. A 2017 study closely investigated the role of the MMR pathway in *C. neoformans* by deleting *MSH2, MLH1*, and *PMS1* and making double mutants of each strain [114]. The study observed that deletions in the MMR pathway led to rapid microevolution and rapid resistance to antifungal agents. Interestingly, the deletion mutants for the MMR pathway also had a different profile of mutations compared with wild type, showing an increase in both transition mutations and single nucleotide insertions and deletions occurring in homopolymeric tracts. In contrast with previous work, deletions in *MLH1* and *MSH2* did not cause any changes in virulence compared with wild type [114,115]. Mutations in the MMR pathway cause an increase in 200-fold in rate of mutations compared with wild type, suggesting a mechanism for rapid microevolution in *C. neoformans* [114]. WGS of relapse isolates have revealed SNPs in *MSH2*, perhaps due to the increased drug resistance caused by that mutation [94]. A higher rate of microevolution has also been observed in *C. deneoformans* strains that have a mutation in *POL3*, a gene that encodes for the DNA polymerase Δ subunit [117,118]. Thus far, two independent pathways have been identified in the *C. neoformans* species complex for the development of mutator phenotypes. These mutators are able to rapidly adapt resistance to antifungal drugs, in a way that is less harmful to fungal cell fitness than aneuploidy. Mutators are also able to quickly develop new phenotypes (Figure 4B) [114]. Though they do not seem to have improved virulence compared with wild type, future studies may reveal that *C. neoformans* isolates with mutator phenotypes are able to more quickly adapt to the host environment.

As mentioned earlier, titan cells are enlarged cells that arise during the initial pulmonary infection. In the lungs, 20–30% of *C. neoformans* cells convert into titan cells [64]. While *C. neoformans* is primarily a haploid yeast consisting of one set of 14 chromosomes, titan cells are polyploid [64]. Despite their increased size and ploidy, titan cells are able to bud and undergo cytokinesis to produce typical-sized daughter cells with reduced ploidy [76]. Gerstein et al. showed that titans are capable of generating haploid and aneuploid daughter cell populations *in vitro* that exhibit increased resistance to fluconazole, oxidative, and nitrosative stress (Figure 4C) [76]. Aneuploid formation underlying fluconazole resistance is well documented in *C. neoformans* and was recently shown to occur during fluconazole treatment in human infections [119,120]. Aneuploidy is often thought to be detrimental to an organism’s fitness, but under certain conditions, especially during times of stress, aneuploidy may be beneficial [121]. The finding that titan cells are able to produce aneuploid populations suggests they may act as a source of rapid adaptation during infection (Figure 4C). Further analysis of the genomic changes produced by titan cells *in vivo* is necessary to better understand the contribution of titan cells to host adaptation and provide further insight into the genomic changes that are important for survival in the host.

In this section, we summarized three potential mechanisms underlying microevolution in *C. neoformans* that result in DNA alterations. It is important to note that changes in the regulation of genes important to survival and host adaptation are not limited to genetic alterations. Epigenetic modifications can also produce rapid changes in gene expression. These modifications and subsequent transcriptome changes likely also facilitate host adaptation in *C. neoformans*. Previous studies have shown that chromatin remodeling controlled by histone deacetylases results in changes to virulence phenotypes [122,123] and the post-transcriptional process of mRNA decay also plays a critical role in stress response and thermotolerance [124].

## Concluding remarks

Historically, studies on the biology and genetics of the *Cryptococcus* sp. have largely been performed independently from clinical studies. Yet, recent translational studies have highlighted the importance of the genotype and phenotype of *C. neoformans* strains to clinical outcome in patients. These studies have uncovered critical gaps in our understanding of how *C. neoformans* and the other species within the *Cryptococcus* species complex adapt to and cause disease within the host. Future research needs to focus on better understanding of the host–pathogen interaction, development of useful models that accurately recapitulate human disease phenotypes, and a better understanding of the path from genetic variation to phenotypic variation and ultimately disease characteristics of the *Cryptococcus* species.

## Abbreviations

CSF: cerebrospinal fluid
GWAS: genome-wide association study
INDEL: insertion/deletion
LD_50_: lethal dose for 50% of mice
MLST: multilocus sequence typing
MMR: mismatch repair
SNP: single nucleotide polymorphism
ST: sequence type
TE: transposable element
WGS: whole-genome sequencing
